RETRACTED

# Evaluation of 3D surface scanners for skin documentation in forensic medicine: comparison of benchmark surfaces

**DOI:** 10.1186/1471-2342-7-1

**Published:** 2007-01-31

**Authors:** Wolf Schweitzer, Martin Häusler, Walter Bär, Michael Schaepman

**Affiliations:** 1 Institut für Rechtsmedizin, Universität Zürich, Zürich, Switzerland; 2 Centre for Geo-Information, Department of Environmental Sciences, Wageningen University, The Netherlands

## Abstract

**Background:**

Two 3D surface scanners using collimated light patterns were evaluated in a new application domain: to document details of surfaces similar to the ones encountered in forensic skin pathology. Since these scanners have not been specifically designed for forensic skin pathology, we tested their performance under practical constraints in an application domain that is to be considered new.

**Methods:**

Two solid benchmark objects containing relevant features were used to compare two 3D surface scanners: the ATOS-II (GOM, Germany) and the QTSculptor (Polygon Technology, Germany). Both scanners were used to capture and process data within a limited amount of time, whereas point-and-click editing was not allowed. We conducted (a) a qualitative appreciation of setup, handling and resulting 3D data, (b) an experimental subjective evaluation of matching 3D data versus photos of benchmark object regions by a number of 12 judges who were forced to state their preference for either of the two scanners, and (c) a quantitative characterization of both 3D data sets comparing 220 single surface areas with the real benchmark objects in order to determine the recognition rate's possible dependency on feature size and geometry.

**Results:**

The QTSculptor generated significantly better 3D data in both qualitative tests (a, b) that we had conducted, possibly because of a higher lateral point resolution; statistical evaluation (c) showed that the QTSculptor-generated data allowed the discrimination of features as little as 0.3 mm, whereas ATOS-II-generated data allowed for discrimination of features sized not smaller than 1.2 mm.

**Conclusion:**

It is particularly important to conduct specific benchmark tests if devices are brought into new application domains they were not specifically designed for; using a realistic test featuring forensic skin pathology features, QT Sculptor-generated data quantitatively exceeded manufacturer's specifications, whereas ATOS-II-generated data was within the limits of the manufacturer's specifications. When designing practically constrained specific tests, benchmark objects should be designed to contain features relevant for the application domain. As costs for 3D scanner hardware, software and data analysis can be hundred times as high compared to high-resolution digital photography equipment, independent user driven evaluation of such systems is paramount.

RETRACTED

**Index terms:**

Forensic pathology, Rough surfaces, Surface Scanning, Technology Assessment

## 1. Background

Courts typically rely on forensic pathologists to document injuries or skin conditions for the purpose of negotiating interpretation and legal significance. During these deliberations, newly raised hypotheses may require details not documented initially. Usually by the time a court trial opens, concerned deceased are buried or cremated and injuries of living people have healed – so the originals are never present any more. Skin surfaces featuring injuries can be fully digitized to be able to conduct a detailed re-analysis, but success relies on precise representation of injured skin.

Other applications of precisely digitized surfaces in forensic pathology include the attempt to reconstructive juxtapositioning [1,2], facial [3] or dental [4] landmark projection for the purpose of quantifying shape match or non-match.

However, most 3D surface scanners are not optimized for injured skin but for industrial or technical application domains such as industrial design, reverse engineering and rapid prototyping. Surfaces typically contain smooth and mostly straight or curved surfaces joined by edges or bends, holes, slots, pockets or grooves [5], which is reflected in the range of test objects used for industrial scanner evaluation [6]. For the purpose of surface scanning, spray paint may be used to reduce artifacts originating from specular reflectance, directional effects, or even discoloration.

In contrast, forensic pathology of injured skin deals with complex, differently colored, locally highly reflective and small sized surface features that may still contain forensic relevance when smaller than 1 mm. We evaluated current 3D surface scanner technology for routine 3D skin surface documentation in forensic pathology, an application domain the scanners that we evaluated were not specifically designed for.

The benchmark problem we posed was whether a 3D surface scanner could capture a whole body including skin findings as small as a needle mark (typically sized 0.5 – 1.0 mm) in a device setting typical for digitizing whole body surfaces within a short amount of time. We base this requirement on our observation that many forensic case re-evaluations focus on small (rather than large) findings, and are conducted at a time when a body has been cremated or buried or when wounds have been changed by surgical treatment or healing. We devised two benchmark objects to match these practical requirements.

RETRACTED

This paper reports handling, usage and 3D scan data comparison of our benchmark objects under practical constraints.

## 2. Methods

### A. Choice of scanners

Choice of scanners was reduced by eliminating models clearly not suitable for the task first: upon visiting an international industry exhibition (Euromold, Frankfurt), an exhaustive internet search and visits to representatives oft two companies for preliminary field tests, all but two surface scanners were either declared to yield or effectively yielded a strikingly insufficient performance for the benchmark problem. These two devices were subsequently tested: The ATOS-II by GOM (Braunschweig, Germany), and the QTSculptor by Polygon Technology (Darmstadt, Germany).

### B. Benchmark objects

Stability is a hard requirement for benchmark testing, so we used two [7] solid benchmark objects not subject to decay: the surface of the nasofrontal bones of a sheep skull and a washed sandstone conglomerate with quartz inclusions (Fig. 1). Realistic skin samples had been considered for scanner evaluation, but were not used because they were subject to considerable intra-object variation in their appearance and did not provide any stable 3D geometry (see Fig. 2).

**Figure 1:** Benchmark objects used: Left: Photo of a sheep's skull containing small intrinsic bone surface features and tool marks, including add-ons such as boreholes, countersink drillings, red and black felt pen marks. Right: Photo of a sandstone conglomerate featuring different inclusions, some of dark light absorbing quality, some highly reflective.

**Figure 2:** Skin sample (pig skin from an animal killed for nutritional purposes) illustrating the non-suitability of realistic skin samples for benchmarking 3D scanner resolution for rough surfaces. Photographs showing decay 3 days (a) and 6 days (b) post mortem. QTSculptor derived 3D surface scans at 3 days (c) and 6 days (d) (bar 1 cm) post mortem provide surfaces of similar appearance, but even at good overlap positioning a distance map (e) between the two digitized surfaces shows they are not congruent with patches of divergence exceeding 2 mm.

Both objects were selected and additionally modified with countersink drillings, boreholes, scratches, and felt pen marks so they would contain a range of challenging shape features typically encountered in forensic skin pathology such as fractal granularity or roughness, holes, scratches, highly reflective patches, shape convexity matching ears, hand or feet as well as discoloration. Typical features in forensic skin pathology include superficial or deep abrasions that may contain highly reflective regions such as body fluids or attached material such as gravel (Fig. 3a/3b), injuries such as gunshot wounds  (Fig. 3d/3e) as well as stab wounds caused by knife blades with by serrated (Fig. 3g) or straight (Fig. 3h) edges.

RETRACTED

**Figure 3:** Side-by-side comparison of real forensic skin pathology (a, b, d, e, g, h) and benchmark object features (c, f, i): Deep facial abrasion after sliding over a rough surface (a, b) containing various highly reflective surface regions, patchy dark discoloration as well as bumpy appearance. These surface shape elements are represented on a similar scale on the rock surface that we used as benchmark object (c). Superficial abrasions as found in gunshot entry wounds (d, e: arrow) are also present on skull surface (f: arrow) used as benchmark object. Curved (g: arrow) and straight (h: arrow) wound edges as found in stabs from a serrated (g) or straight (h) knife blade are represented by a bony suture of the skull (i: arrow) used as benchmark object (bar 1 cm).

### C. 3D scanners and data acquisition

Both scanners projected collimated white light patterns for optical triangulation and manufacturers' declared specifications did not differ significantly (Table 1). Calibrations were performed using patterned calibration targets. Scans were obtained in a stationary setting without particular vibration isolation, but no vibration was incurred during the scans.

**Table 1:** Device and setup parameters of the two surface scanners

Specification/parameter [*: according to manufacturers' specification]	ATOSII	QT-Sculptor PT-M1280
Measuring distance/Stand off used for benchmark scans	about 75 cm	about 80 cm
Measuring volume *	100 × 80 × 80 mm^3^	120 × 100 × 100 mm^3^
Camera resolution *	1280 × 1024 pixel	1280 × 960 pixel
Lateral point spacing *	0.08 mm	0.08 mm
Noise (depth) *	0.002 mm	0.015 mm

Both scanners require objects to be captured from different directions and for this test, objects were placed on a turning table and 8 – 12 single scans were acquired. Automatic image merging for 3D surface model generation, which was done subsequentially, required reference point stickers to be placed on objects only for the ATOS-II scanner prior to the scan but not for QTSculptor. Software control of scanner was integrated with computer hardware and subsequent scan image registration was based on particular file formats for both devices. This is why we evaluated each hardware-software package sold as "3D scanner" in conjunction.

The ATOS-II used for this evaluation was owned by a local government department and operated by a professional who had completed a considerable number of scans. The QTSculptor PT-M1280 was tested by a novice on the manufacturer's premises. The nature of the benchmark test had been declared to the investigators prior to the scans.

RETRACTED

We proceeded to compare resulting 3D data without further manual point-click editing of the data which – as opposed to mathematical operations applied to whole images – could be viewed as tampering with visual evidence in forensic sciences. Relevant differences pertaining to duration of worksteps are contained in Table 2.

**Table 2:** Scanner handling

Work step	ATOSII	QT-Sculptor
Special setup of object surface	Requires reference point stickers to be placed on object ~ 5 min	not required
Approximate user attended scan time for skull benchmark object	~ 15 min	~ 8 min
Approximate user attended scan time for rock benchmark object (difficulty: convex object).	~ 30 min	~ 12 min
Post processing of data		~ 5 – 15 min
Rock: Number of polygons	5,005,559	3,556,544
Skull: Number of polygons	4,430,998	2,447,596

### D. 3D data rendering and photographs

3D data was surface-rendered using a non-texturized gray surface structure, oblique virtual illumination and orthogonal projection (see Figures 4, 5, 6 and 7). Resulting 2D projections (best rendering resolution 10–20 μm) were complemented with similarly illuminated digital microscopy photographs of matching object surface areas (best resolution 10–20 μm). Only surfaces and no textures were processed.

**Figure 4:** Sheep skull benchmark object. a): Photo. b) Matching the photo, this shows the 3D model obtained using ATOS-II 3D scanner. c) Matching the photo, this shows the 3D model obtained using QTSculptor scanner. Details of the scratch contained on the surface were reproduced photographically (d), on the ATOS-II scanner (e) and QTSculptor (f). See text for feature description. Bar is 5 mm.

**Figure 5:** Rock benchmark object. a): Photo. b) Matching the photo, this shows the 3D model obtained using ATOS-II 3D scanner. c) Matching the photo, this shows the 3D model obtained using QTSculptor scanner. A detailed region of this surface was reproduced photographically (d), on the ATOS-II scanner (e) and QTSculptor (f). See text for feature description. Bar is 5 mm.

**Figure 6:** Experimental subjective evaluation was conducted using a set of 20 comparisons just as the three visual objects (a, b, c) displayed here, evaluated by 12 participants. For each of the rows, scanner 'x' and scanner 'y' were presented in random sequence to participants who had to select the preferred match ('x' or 'y') as a forced choice. In this illustration, 'x' is QTSculptor, 'y' is ATOS-II for all three visual objects (a,b,c). a: Bone surface structure featuring finely granular roughness, and sharp edges (bottom of foramen), that blend into the surface (lateral margins of the foramen). b: Bone surface structure featuring finely granular roughness, a black felt pen dot, several small surface indents, and a suture. c: Bone surface containing a more extensive suture containing countersink drillings. Bar is 5 mm.

RETRACTED

**Figure 7:** Quantitative characterization of scanner performance was done using a set of 220 single surface areas, 3 of which are presented for illustration with photos of real object (a,d,g), ATOS-II-derived data (b,e,h) and QTSculptor-derived data (c,f,i). Red outlines mark homologue areas. Bar is 5 mm.

### E. Experimental subjective evaluation

In a comparison experiment, we presented a test set containing 20 different visual objects to 12 participants: one photo of a portion of a benchmark object, and two matching images with rendered 3D data randomly placed to the left (X) or right (Y) (see Fig. 6 for illustration of 3 instances of the 20 objects). Of the 12 participants, 10 were professionally occupied with shapes (9 in forensic pathology, 1 in industrial tooling), 2 were not working with shapes (clinical researchers). None was directly involved with this study. For each of the 20 objects, participants had to indicate which scanner-derived image better matched the photo in a forced choice. A total of 240 (12 × 20) answers resulted.

### F. Quantitative characterization of 3D data

In optical triangulation of rough surfaces using light patterns, uncertainties at each image pixel significantly depend on illumination and measurement angles at that precise location. On rough surfaces, this angle varies from one point in the original single image to the next, and so does the accuracy and sensitivity of the surface scanning system; at an extreme, the system may have no sensitivity at all for some image patches, whereas neighboring image patches may exhibit higher local accuracy and contribute to a correct overall appearance of the resulting digital surface [8]. This means, that in order to appreciate the quality of digitized rough surfaces, the inherent nature of the error requires single small regions or patches to be checked individually.

We conceptually decomposed the scanned surface data (y) into a match of the ideal real object (μ) with additional deviating features (e) [9]:

*y*_*scanner *_= μ_*object *_+ *e*_*deviating_features *_[Eq.1]

We expected the deviation of the surface data from the benchmark object to be possibly dependent on the minimal extent (s) and appearance (a) of shape elements [10].

*e*_*deviating_features *_= *f*(*s*,*a*) [Eq.2]

Currently, macroscopic and microscopic inspection, including subsequent verbalization and categorization of observations, is the only technique yielding sufficient accuracy that is recognized as *de-facto *standard in forensic pathology. Any automatic method eligible as reference would have to be suitably accurate with a ratio of 10:1 over the method tested [11] (any lower ratios may be regarded as concession to manufacturers), and so far, no automated 3D surface digitizer was established either as reference method or accepted as standard method in forensic skin pathology by any authority.

RETRACTED

Across both benchmark objects, 220 single surface patches in the lower range of the visual scale containing distinct features were selected arbitrarily, labeled, categorized, and their smallest spatial extent was measured directly on the object using a micrometer.

As a minimum of five different surface materials are required [9], surface patches were classified on the macerated skull as (a) native surface, (b) black discoloration and (c) red discoloration, and on the sandstone as (d) rough surface and (e) quartz inclusion. Shape elements were categorized as (i) granular 3D texture versus directional or streak 3d texture and (ii) repetitively monotonous versus non-repetitively sparse structures [12].

Projected 3D-appearances of homologue single surface areas of each of the two scanners were awarded binary scores as to whether they constituted a sufficient representation or not upon direct comparison with the benchmark object (illustrated in Fig. 7). Based on this, data of each 3D scanner was independently awarded a "1" for sufficiently and a "0" for insufficiently representing a particular surface area. Recognition rates were obtained by totaling these counts.

Conceptual problems with confidence intervals of binary scores [13] were avoided by analysing a completely stratified dataset. Bootstrap [14] was used to determine confidence intervals.

Recognition rates were correlated with size and surface categories (Tables 3 and 4) using the Chi-Square test. Logistic regression can determine continuously varying recognition rates from categorized data and was used to determine how recognition rates would continuously degrade with diminishing feature size (Fig. 8; significance levels see Table 4).

**Table 3:** Quantitative characterization of 3D data with respect to recognition rate

Items compared	ATOSII	QTSculptor	Statistics
Total surface area count recognized/not recognized on scanner data	114/106	212/8	p < 0.001 χ^2^
Recognition rate Cat. A > 0.7 mm	66/19	85/0	p < 0.001 χ^2^
Recognition rate Cat. B ≤ 0.7 mm	48/87	127/8	p < 0.001 χ^2^
Recognition rate (bootstrapped estimate)	73 ± 5% @ ≥ 1.2 mm	98 ± 1% @ ≥ 0.3 mm	
*Surface categories*	*Recognized/not recognized:*	*Recognized/not recognized:*	
Bone native surface	43/36	77/2	p < 0.001 χ^2^
Black dots on bone surface	4/1	5/0	
Red dots on bone surface	1/1	2/0	
Sandstone surface	66/61	121/6	
Quartz inclusion (highly reflective)	0/7	7/0	

RETRACTED

**Table 4:** Size dependency of recognition rate

Scanner model	Smallest feature extent [mm] – recognized	Smallest feature extent [mm] – not recognized	Statistical significance (Chi Square) for fit of logistic regression model (Fig. 6)
ATOSII	0.96 ± 0.71 mm *logarithmic transform: -0.3 ± 0.8 mm*	0.47 ± 0.75 mm *logarithmic transform: -1.4 ± 1.0 mm*	p < 0.0001
QTSculptor	0.74 ± 0.77[*] mm *logarithmic transform: -0.8 ± 1.0[#] mm*	0.28 ± 0.24[*] mm *logarithmic transform: -1.7 ± 1.0[#] mm*	p < 0.0183

**Figure 8:** Logistic regression model fit for smallest feature size (x-axis) against recognition rate for ATOS-II scanner (left) and QTSculptor scanner (right).

Heteroscedastic data – i.e., data exhibiting unequal variances between groups – is assumed to yield reduced significance for statistical tests if variances are truly different; however, what appeared to be initially unequal variances was a result of differently scaled data and thus rendered homoscedastic by using a logarithmic transform [15].

### G. Statistics, visualization and computer hardware

Benchmark objects were photographed using a digital consumer camera (Finepix F610, Fuji Photo Film Co. Ltd., Tokyo, Japan) and a microscope-mounted (Wild M3Z, Leica-Microsystems, Glattbrugg, Switzerland) scanner camera (Progres, Jenoptik, Germany). 3D surface data was processed and visualized using IDL (Interactive Data Language, Research Systems Inc., Boulder, CO, USA) on a workstation (Intellistation 275, International Business Machines IBM, White Plains, NY, USA). Statistical computations were performed using the software packages JMP (SAS Institute Inc., Cary, NC, USA) and SYSTAT (Systat Software, Inc., Point Richmond, CA, USA).

## 3. Results

### A. Setup and handling

Both scanners provided a straightforward overall approach to object setup and handling. Some reference point stickers required by the ATOS-II fell off without apparent reason, and were replaced before the scan, but not during the scan procedure. Total time requiring user attendance was less than half the time on the QTSculptor scanner than on the ATOS-II scanner. ATOS-II generated considerably larger 3D models than the QTSculptor (Table 2).

### B. Qualitative appreciation and individual details

Qualitatively (Figure references in brackets), similarities and differences of scanner generated data can be appreciated by comparing photographs (4a, 4d, 5a, 5d, 6/photo, 7a, 7d, 7g) with matching scan data of ATOS-II (4b, 4e, 5b, 5e, 6/Y, 7b, 7e, 7h) and QTSculptor (4c, 4f, 5c, 5f, 6/X, 7c, 7f, 7i).

RETRACTED

While the overall appearance of both scanner's data seems to match the original object at first glance, individual surface patches exhibit discernible differences: A bone surface scratch lacks details on the ATOS-II generated surface (4b/1, 4e/1) but is well discernible on QTSculptor derived data (4c/1, 4f/1). The roughness of the finely granular bone surface (4a/3, 6a/photo, 7d) appears to be adequately represented on QTSculptor generated data (4c/3, 6a/X, 7f) but not on the surface documented with ATOS-II (4b/3, 6a/Y, 7e), where a markedly less granular structure is exhibited. Slightly more coarsely granular surface (6c/photo, 7g) exhibits defects on ATOS-II (6c/Y, 7h) but not on QTSculptor (6c/X, 7i). Small grooves present on the sandstone rock (5a/1, 5d/3: between arrows; 7a) are discernible on QTSculptor derived data (5c/1, 5f/3: between arrows; 7c) but not on the ATOS-II generated surface (5b/1, 5e/3; 7b); two distinct humps present on the rock (5a/2: arrows) can be differentiated on QTSculptor data (5c/2) but not on the data off the ATOS-II scanner (5b/2) where that distinction is blurred. Borehole rims (4a/2) are available for inspection in QTSculptor data (4c/2) but not on ATOS-II derived data (4c/2). Black patches (6b/photo) seem to cause the ATOS-II to represent a hole (6b/Y), whereas the QTSculptor contains a surface patch (6b/X). Shiny quartz inclusions (5a/4, 5d/5) lead to defective surface data under the ATOS-II scanner (5b/4, 5e/5) but not when scanned with QTSculptor (5c/4, 5f/5). Furthermore, ATOS-II generated surface contains some shape information not present on the object; correlates for these are locations of reference point stickers (4b/4, 5b/7, 7b).

Overall the ATOS-II generated surfaces contain more details, better representation of highly reflective and finely granular rough surfaces, better representation of dark surface regions, and more surface attached to holes.

### C. Experimental subjective evaluation

For each of the 12 individual test sets, a total of 20 votes per test set yielded an average of 17.3 ± 2.2 (min: 13/20, max: 20/20) in favor of QTSculptor generated data. In all 240 answers obtained by forced choice, 208 (87.0 ± 3.4%) votes were issued for QTSculptor generated data which is significantly more than the 32 (13.0 ± 3.4%) votes yielded by ATOS-II generated visual objects (bootstrapped standard deviation using 2000 re-samples of the size n = 100 (out of 240); p < 0.0001, Wilcoxon nonparametric test).

### D. Quantitative characterization of 3D data

Smallest spatial extent of the 220 features used for this characterization contained in a median of 0.5 mm (25th percentile at 0.2 mm, 75th percentile at 1.0 mm). Overall recognition rate as well as recognition rate for each of the two groups – category A > 0.7 mm and category B ≤ 0.7 mm – was significantly better for QTSculptor (χ^2^: p < 0.001) (Table 3).

RETRACTED

Logistic regression (see Fig. 8 and Table 4) showed that recognition rate was over 90% for features at least 0.3 mm in smallest extent in the QTSculptor (Table 4: * original data with unequal variances; #: homoscedastic data after logarithmic transform). Bootstrapped recognition rate estimate for QTSculptor was 98 ± 1% for features minimally sized ≥ 0.3 mm (2000 resamples with resample size = 100). On ATOS-II generated data, logistic regression revealed a recognition rate of over 70% for surface areas at least 1.2 mm in size and bootstrapped recognition rate estimate was 73 ± 5% for features minimally sized ≥ 1.2 mm (2000 resamples with resample size = 100).

Classification of 220 single surface areas yielded 79 bone surface areas, 5 bone surface areas with black discoloration, 2 bone surface areas with red discoloration, 127 sandstone and 7 quartz inclusion areas. The shape elements contained were 176 granular, 27 directional, 17 complex; patterns observed were 182 non-repetitive and 38 repetitive. No geometric characteristic (repetitive, non-repetitive; granular, directional, complex) caused significant differences in recognition rates between both scanners tested. In particular, directional shapes (such as scratches) and granular shapes (such as little indents, protrusions or rough patches) did not yield significantly different recognition rates. The ATOS-II scanner showed difficulty in digitizing highly reflective (sandstone quartz inclusions) or discolored (red, black) surface regions.

Three examples representative of the total of the 220 instances that we analyzed are shown in Fig. 7: A groove on the rock (Fig. 7a) is visualized on QTSculptor data (Fig. 7c), but not on ATOS-II data (Fig. 7b). Fine granularity of rough surface (Fig. 7d) was adequately matched in data by QTSculptor (Fig. 7f) but not ATOS-II (Fig. 7e). Presence of a little ditch (Fig. 7g) could be visually discerned on data by QTSculptor (Fig. 7i) but not by ATOS-II (Fig. 7h).

## 4. Discussion

Realistic tissue samples showed to be unreliable for benchmarking 3D scanners as decay and plasticity cause skin to exhibit varying 3D shapes. Instead, we used two solid benchmark objects that contained representative geometric aspects of relevant forensic skin pathology (Fig. 3).

The targeted purpose of digitized documentation determines the means employed [16]: Is a scanner merely used to 'add a flavor of 3D'? Is 3D data obtained to examine new hypotheses for further investigation? Is data collected to confidently certify the absence of relevant injuries at a later point in time?

RETRACTED

Controversial or discriminating morphology may appear small to the naked eye and can be easily overlooked. Such injuries may include hard to detect needle-marks that raise suspicion of poisoning [17], tentative cuts which may indicate self infliction [18] or soot patterns that are important for drawing conclusions about weapon, ammunition and shooting range [19-21]. Those injuries define the size range that should be captured by a 3D scanner in order to allow for a later re-analysis of a case.

Conversely, technical constraints of surface scanners intrinsically link higher resolution with a smaller field of view, and therefore a longer total scan time. That is why we tested 3D scanner performance under practical constraints, focusing on 'smallest possibly important feature' combined with 'usefully short amount of time'.

Our tests show conclusively that the surface scanner QTSculptor performs faster and obtains significantly better results in the context of relevant medico-legal skin surface documentation despite similar manufacturers' specifications. User attended time to operate the scanners was about double for the ATOS-II, and generated ATOS-II data was considerably larger. We acknowledge that results of constrained tests may differ considerably from a theoretical optimum: given unlimited time and user attendance, the ATOS-II scanner may also achieve acceptable results on rough surfaces.

Any digitized data requires a minimal resolution of 16 to 24 data elements in each dimension (pixel, voxel, 3D coordinate points) for an adequate representation of a real feature [22] while a resolution of 50 to 60 elements per feature would be a good resolution. Based on a quantitative analysis, smallest feature sizes that are documented by the QTSculptor ranged down to 0.3 mm for around 98.1%, pointing to an effective lateral 3D point resolution in the range of 15 to 20 μ (noise 2 μ according to manufacturer). Conversely, the ATOS-II managed to capture features sized as small as 1.2 mm in around 70%, pointing to an effective lateral 3D point resolution around 60 μ (noise 15 μ according to manufacturer). Both manufacturers declared a lateral point spacing of 80μ. The ATOS-II matched its manufacturer's specification as to resolution in this test while the QTSculptor obviously exceeds it. This would be hard to establish using automated methods: simple computable data classifiers such as mean square error only provide poor correlation with visually perceivable image quality [23].

Higher effective resolution of the QTSculptor is also indicated by the better representation of fine granularity, observed on digitized rough surfaces; a coarser grain contained in matching ATOS-II generated data indicates aliasing as a result of sub-Nyquist sampling frequency, i.e. undersampling or insufficient resolution in relation to the structure under study [24,25]. The better representation of rough surfaces, rims of boreholes and bottom regions of countersink drillings, and the faster and better acquisition of the convex and rough rock surface also indicate a better depth-of-field of the QTSculptor.

RETRACTED

Experimental subjective evaluation of the surface samples by 12 judges conclusively showed that 3D surface generation of the QTSculptor is significantly superior compared to the ATOS-II. It is known that subjective evaluation is fast and highly effective [26] and reliability increases with the number of judges; a reliability rating of 0.90 can be obtained with 10 – 50 judges [27]. This subjective evaluation matched the result of other modes of comparison that we had employed, and using projected 2D imagery seemed to be important. In evaluating 3D methods, one may have to exert specific caution not to expose oneself too much to interactive displays: 3D appearance may cause a person to perceive the quality of a 3D model as better when interactively manipulating data on a fast computer compared to its static 2D appearance [28].

Technical flaws in the surfaces obtained by the ATOS-II scanner included reference point stickers that not only created round bumps on the digitized 3D surface, but also, covered up object surface underneath. One could justify using reference stickers if they would cause the result to be of greater accuracy or if the scan process would progress significantly faster due to these stickers. Systems using point stickers might perform better in slight moving or not full stable target conditions; yet the ATOS-II scanner neither produced results of greater accuracy nor did it exceed the speed of the data capture process of the QTSculptor.

An important reason for the ATOS-II scanner being outperformed by the significantly cheaper QTSculptor may be the application domain it is specifically designed for – industrial surface scanning. There, reference point sticker based methods may outperform any other 3D method in terms of accurately and precisely placing single 3D coordinates in data space while safely interpolating points in between – yet that was not the output required in this benchmark test. In fact, manufacturer's specification of what is or is not accurate may not coincide with any particular application's requirement for accuracy.

Theoretical advantages of high-quality digital 3D-documentation include the option of examining complex 3D shapes from close-up at any later point in time without the limitation of depth-of-field, always producing focused 2D-imagery. This limitation of real photography cannot be overcome even by employing latest technology such as a plenoptic camera [29].

RETRACTED

## 5. Conclusion

We have shown that despite similar manufacturers' specifications, one 3D scanner (QTSculptor) significantly outperformed another model (ATOS-II) both quantitatively and qualitatively under practical constraints in a specific benchmark test that was devised for an application domain neither of the two scanners had been specifically designed for – forensic skin pathology.

As costs for 3D scanner hardware, software and data analysis can be hundred times as high compared to high-resolution digital photography equipment, independent user driven evaluation of such systems is paramount.

## Competing interests

The author(s) declare that they have no competing interests.

## Authors' contributions

MH and WS both practically organized and supervised the benchmark testing and discussed ideas to write up the manuscript. WS planned the study, carried out the design of the test and the benchmark objects, studied relevant literature, analysed the resulting data, documented the figures, conducted the statistics and wrote the manuscript. WB and MS contributed to the content of the manuscript. All authors read and approved the final manuscript.

## Pre-publication history

The pre-publication history for this paper can be accessed here:


